The article "Effect of Rituximab on 24-Hour Urine Protein and Albumin or Renal Function in Patients with Glomerulonephritis" was retracted in 2023. Reasons: suspected computer-generated content; unreliable results or conclusions; lack of ethics approval or compliance; missing or withdrawn patient consent.

# Effect of Rituximab on 24-Hour Urine Protein and Albumin or Renal Function in Patients with Glomerulonephritis

**DOI:** 10.1155/2022/6412740

**Published:** 2022-04-13

**Authors:** Fangzhong Huang, Jian Huang, Yan Liu, Jinli Li

**Affiliations:** Jinhua Municipal Central Hospital (Affiliated Jinhua Hospital, School of Medicine, Zhejiang University), Jinhua 321000, Zhejiang, China

## Abstract

This study aimed to investigate the correlation between the urine protein/creatinine ratio (PCR) and 24 h urine total protein quantity (24hUTP) in morning and random urine and its prediction equation. Rituximab (RTX), a monoclonal antibody that acts on the B cell epitope CD20, has been used in the renal field since 2005 and has become a hot topic in the clinical treatment of many glomerulonephritis diseases. Apart from focusing on the safety and efficacy of RTX in clinical treatment, some scholars are still working on the mechanism of its action in the treatment of renal diseases, trying to find its specific targets in renal tissues. *Results*. There was no significant difference between morning urine PCR, random urine PCR, and 24hUTP (*P*=0.81); there was a significant positive correlation between morning urine PCR and 24hUTP (*r* = 0.90, *P* < 0.01) and between random urine PCR and 24hUTP (*r* = 0.95, *P* < 0.01), and the correlation between random urine PCR and 24hUTP was higher than that between morning urine PCR and 24hUTP. The results of the ROC curve analysis showed that the correlation between morning urine PCR, random urine PCR, and 24hUTP was higher than that between morning urine PCR and 24hUTP in different groups. The optimal threshold values for random urine PCR to predict 2.4hUTP were 0.56 g/g (sensitivity 93.5%; specificity 75.4%), 1.11 g/g (sensitivity 98.3%; specificity 92.4%), and 3.43 g/g (sensitivity 87.9%; specificity 89.9%), respectively. The equations for predicting 24hUTP by morning urine PCR and random urine PCR were as follows: (1) 24hUTP(g) = 0.793 + 0.793 × morning urine PCR + 0.124 × total cholesterol − 0.177 × Alb (coefficient of determination *R*^2^ = 0.87); (2) 24hUTP(g) = 0.369 + 0.856 × random urine PCR + 0.132 × total cholesterol − 0.092 × Alb (coefficient of determination *R*^2^ = 0.92); the prediction equation of random urine was more accurate than that of morning urine. The correlation was not affected by gender, age, 24 h urine volume, etiology, eGFR, Alb, or total cholesterol level, and the correlation between random urine PCR and 24hUTP was higher than that of morning urine PCR. CR prediction equation was used instead of the 24hUTP test.

## 1. Introduction

Focal segmental glomerulosclerosis (FSGS) is a common type of glomerulonephritis. Gunnarsson et al. [1] have found that the annual incidence of FSGS is (0.2–1.8) per 100,000 globally, while a 12-year study in the USA showed that FSGS was the most common type of pathology on renal biopsy (approximately 39% of cases). According to the Kidney Disease: Improving Global Outcomes (KDIGO) guidelines, the current first-line treatment options for FSGS include angiotensin-converting enzyme inhibitor (ACEI), haemodialysis inhibitor (HTA), anaerobic syndrome (ASA), angiotensin II receptor blocker (ARB), hormones, and immunosuppressants [2]. However, patients with steroid-dependent nephrotic syndrome (SDNS) are more likely to experience adverse effects with either long-term hormone therapy alone or hormone therapy combined with immunosuppressant therapy, and in the case of steroid-resistant nephrotic syndrome (SDNS), patients are more likely to experience adverse effects with hormone therapy [3]. In patients with steroid-resistant nephrotic syndrome (SRNS), not only is hormone therapy alone ineffective but some patients do not achieve clinical remission despite the addition of immunosuppressive drugs. Therefore, the search for new treatment options for FSGS has become one of the hot topics of research in China and abroad [4].

RTX, a human-mouse chimeric monoclonal antibody acting on the B cell epitope CD20, has been approved by the Food and Drug Administration (FDA) for use in non-Hodgkin's lymphoma, chronic lymphocytic leukemia, rheumatoid arthritis, and antineutrophil cytoplasmic antibodies [5]. As an initial therapeutic agent for haematological and autoimmune diseases, RTX has been used for a short time in the treatment of renal diseases, and there is no consensus on the dose and duration of treatment. Lindholm et al. [6] have shown that RTX for FSGS can reduce urinary protein levels in patients, thereby slowing disease progression and protecting renal function. Currently, clinical studies of RTX are mainly found in case reports and single-centre, small-sample retrospective studies, and analyses of large-sample, multicentre randomised controlled trials are lacking [7].

Glomerulonephritis has become one of the major life-threatening diseases and its prevalence is high, with a prevalence of 10.8% among adults in China [8]. The 24-hour urine total protein quantity (24hUTP) is an accepted method for measuring urine protein [9]. However, in practice, this test has many drawbacks in clinical application due to the long retention time, inconvenient urine storage, poor patient compliance, and nonstandard retention process. The NKFK/DOQI guidelines [10] recommend the use of the protein/creatinine ratio (PCR) to determine the total amount of urine protein, and several studies at home and abroad have shown that there is a significant correlation between PCR and 24hUTP.

The PCR has a certain diagnostic value for the determination of urinary protein [11]. In this study, the correlation between morning urine, random urine PCR, and 24hUTP will be analyzed, and a prediction equation will be established to provide a rapid, simple, and accurate means of quantitative assessment of urine protein in clinical work.

## 2. RTX Acts Directly on B Cells for the Therapeutic Effect

RTX acts directly on the B cell epitope CD20 and regulates autoimmunity through three classic pathways of regulation of humoral immunity: apoptosis, complement dependent cytotoxicity (CDC), and antibody-dependent cell-mediated cytotoxicity (ADCC) [12]. CDC and antibody-dependent cell-mediated cytotoxicity (ADCC) are the classical pathways that regulate humoral immunity by reducing the number of B cells and regulating autoimmunity [13]. Among them, in vitro experiments [14] have demonstrated that RTX can directly deplete B cells through CDC or indirectly exert B cell toxicity through the ADCC pathway, which involves a variety of cells, such as natural killer cells, monocytes, and macrophages. Based on long-standing research in basic immunology, it is reasonable to assume that the therapeutic effect of RTX on FSGS, as a monoclonal antibody acting directly on B cells, may be related to its involvement in the B cell-mediated humoral immune response.

CD19 is a common surface marker of B cells, and its expression level directly reflects the level of B cells. Therefore, CD19 is often used clinically as an indicator of the effect of RTX.

In one study [15], RTX was used to treat patients with refractory nephrotic syndrome, and it was found that remission of proteinuria was not equated with the number of B cells; in this study, a single dose of RTX was administered to four children with SRNS (two of whom had been confirmed to have FSGS by renal biopsy). However, at follow-up, the study found that one child relapsed at 4 months with a CD19 level of 0, suggesting that CD19 is not an indicator of the sustained effect of RTX. Subsequently, Colucci et al. [16] investigated the relationship between memory B cells and the effects of RTX and concluded that delayed reconstitution of memory B cells was predictive and protective of relapse in nephrotic syndrome. In this study, 28 children with SDNS/frequent relapsing nephrotic syndrome (FRNS) aged 13.68 ± 0.77 years were enrolled, and the numbers of T and B cell subsets were measured by flow cytometry in SDNS/FRNS children and healthy control children of the same age, including CD19+ B cells (total B cells), transitional B cells, mature B cells, memory B cells, IgM memory B cells, transformed memory cells, CD3+ T cells, CD4+ T cells, and CD8+ T cells. The results showed that SDNS/FRNS children had lower levels of mature B cells (10% vs. 4.5%, *P* < 0.001) and transitional B cells (0.8% vs. 0.3%, *P* < 0.001) and no differences in T cell levels, total B cell levels, and memory B cell levels compared to healthy control children when they had not received RTX treatment [17]. At 1 month after RTX treatment, B cell subsets were suppressed in all 28 children and gradually returned to normal levels in the order of transitional B cells, mature B cells, and memory B cells after 6 months, reaching normal levels at 12 months. The remaining B cell subgroups were also significantly lower at 12 months of treatment than in healthy controls. The 28 children with SDNS/FRNS were followed up for 24 months, with 14 relapsing and 14 not relapsing. A one-way Cox regression model was used to analyse the B cell subsets in the relapsed/nonrelapsed children and showed that the levels of memory B cells, IgM memory B cells, and transformed memory B cells as well as the dose of tacrolimus applied in the past 4 months were all associated with the risk of relapse at 9 months of follow-up. Further multivariate Cox regression analysis found that only the level of transformed memory B cells was significantly associated with the risk of relapse; subject operating characteristic curve analysis showed that the best predictive value for differentiating between relapsed and nonrelapsed children might be the ratio of transformed memory B cells to total lymphocytes [18].

The best predictive value to distinguish between relapsed and nonrelapsed children may be a ratio of transformed memory B cells to total lymphocytes of 0.067% (sensitivity 71%; specificity 93%) or a peripheral blood concentration of 1.65 cells/*μ*L (sensitivity 64%; specificity 86%), i.e., patients with transformed memory B cells/total lymphocytes <0.067% or transformed memory B cells <1.65 cells/*μ*L at 9 months after RTX treatment. The risk of relapse within 24 months was significantly reduced. Thus, transformed memory B cells may be a potential predictor of relapse [19].

Taken together, we have found that most of the research studies on the direct target of RTX, B cells, have focused on the underlying immunological aspects, but there has been no in-depth analysis of the mechanisms of B cell involvement in the remission of proteinuria in FSGS patients. In addition, although FSGS is a common pathological type of nephrotic syndrome and clinical applications suggest that patients with FSGS are well treated with RTX, there is a lack of further subgroup studies on FSGS and other pathological subtypes of nephrotic syndrome. For example, whether there are different mechanisms for RTX in different pathological types of nephrotic syndrome and whether there are different specific indicators for the effect of RTX in different pathological types.

## 3. Study Subjects

Patients selected for consultation at our nephrology department were all eligible for a Western diagnosis of glomerulonephritis and had been ill for >3 months. Exclusion criteria were as follows: those aged <18 years; those with urinary tract infections, haematuria, and acute febrile illnesses; and those with altered urinary protein and blood creatinine (Scr) excretion due to strenuous exercise and female menstrual periods. The study was approved by the hospital ethics committee.

## 4. Methods

### 4.1. Data Collection and Grouping

All patients were given a 2-day dietary guideline based on the dietary criteria for patients with glomerulonephritis. Gender, age, primary disease, estimated glomerular filtration rate (eGFR), Scr, serum albumin (Alb), total cholesterol, and 24 h urine output were collected. Glomerulonephritis was staged according to the clinical guidelines of K/DOQI [20]. The patients were grouped according to Alb, total cholesterol, and 24 h urine output levels.

### 4.2. Sample Collection

#### 4.2.1. Morning Urine

The middle portion of the patient's first urine is collected early in the morning (7:00 a.m.) and used for the morning PCR. 24 h urine: from the time the morning urine is collected, the time is recorded as 7:00 a.m. After this time until 7:00 a.m. the next morning, urine is collected in a graduated container with a preservative (toluene) and the total volume (ml) is recorded. 5 ml of urine is mixed and sent for testing. After mixing, 5 ml of urine was collected and sent for 24hUTP testing.

#### 4.2.2. Random Urine

The urine sample was collected at any time after the morning urine and 24 h urine for random urine PCR.

#### 4.2.3. Blood Samples

Venous blood samples were taken on the day morning urine was collected.

### 4.3. Sample Testing

The samples were tested on a CS-400B biochemical analyzer. Urine protein was measured by immunoturbidimetric Scr, urine creatinine, and total cholesterol by the enzymatic method and serum albumin by the bromocresol green method.

## 5. Results

### 5.1. General Information

A total of 211 eligible patients were included, of whom 107 were males and 104 were females, aged 20–89 years (57.6 ± 16.3 years) (30 cases of diabetic nephropathy, 3 cases of lupus nephritis, and 2 cases of purpura nephritis). Urine samples were collected in 633 cases and blood samples in 211 cases. The results of ANOVA showed that there was no significant difference between morning urine, random urine PCR, and 24hUTP (*F* = 0.21, *P*=0.81); the specific contents are given in Table 1. There was also a significant positive correlation between morning urine PCR and 24hUTP (*r* = 0.90, *P* < 0.01) and a significant positive correlation between random urine PCR and 24hUTP (*r* = 0.95, *P* < 0.01) (Figures 1 and 2).

### 5.2. Correlation between Morning Urine, Random Urine PCR, and 24hUTP in Different Groups

All patients were compared in seven groups according to gender, age, 24 h urine volume, etiology, eGFR, Alb, and total lipid cholesterol. Correlation analysis was performed between morning urine, random urine PCR, and 24hUTP in different groups, and the results showed a positive correlation between PCR and 24hUTP in different groups, with correlation coefficients *r* ranging from 0.50 to 0.99 (all *P* < 0.05). The correlation between random urine PCR and 24hUTP was higher than that of morning urine PCR for all subgroups (Table 2).

### 5.3. ROC Curve

According to the KDIGO guidelines, three different cutoff points for 24hUTP were defined, i.e., 24hUTP ≥ 0.5 g, 24hUTP ≥ 1.0 g, and 24hUTP ≥ 3.5 g. The ROC curves for morning urine PCR and random urine PCR were plotted according to the different cutoff points, as shown in Figures 3–5. The results showed that when 24hUTP ≥ 0.5 g, morning urine PCR ≥ 0.70 g/g was the best diagnostic threshold with an AUC of 0.933 and sensitivity and specificity of 84.4% and 86.0%, respectively; random urine PCR ≥ 0.56 g/g was the best diagnostic threshold with an AUC of 0.957 and sensitivity and specificity of 93.5% and 75.4%, respectively. When 24hUTP ≥ 1.0 g, morning urine PCR ≥ 1.09 g/g was the best diagnostic threshold, with an AUC of 0.987 and sensitivity and specificity of 95.8% and 91.3%, respectively; random urine PCR ≥ 1.11 g/g was the best diagnostic threshold, with an AUC of 0.994 and sensitivity and specificity of 98.3% and 92.4%, respectively. When 24hUTP ≥ 3.5 g, morning urine PCR ≥ 3.81 g/g was the best diagnostic threshold, with an AUC of 0.890 and sensitivity and specificity of 66.7% and 89.9%, respectively; random urine PCR ≥ 3.43 g/g was the best diagnostic threshold, with an AUC of 0.950 and sensitivity and specificity of 87.9% and 89.9%, respectively.

A multiple linear regression analysis was performed with 24hUTP as the dependent variable, morning urine PCR and random urine PCR as independent variables, and age, sex, eGFR, total cholesterol, Alb, and 24 h urine volume as corrected independent variables, as given in Table 3. The results yielded regression equations.

## 6. Discussion

Proteinuria is the most common clinical manifestation in the development and progression of glomerulonephritis and is not only a risk factor for kidney damage but also an independent risk factor for cardiovascular events in patients. It is not only a risk factor for kidney damage but also an independent risk factor for cardiovascular events. Therefore, the quantitative measurement of urine protein is of great importance for the diagnosis, treatment, and prognosis of chronic kidney disease. The 24hUTP test is the gold standard for determining the total amount of urine protein, but the measurement method is complex, the volume of urine collected is highly variable, retention is difficult, and patient compliance is poor. It is also difficult to accurately collect 24 h urine from critically ill patients, children, or outpatients who have difficulty retaining urine. A number of studies have demonstrated that PCR correlates well with 24hUTP, with correlation coefficients ranging from 0.66 to 0.98 and *P* values mostly less than 0.01.

In this study, by analyzing the correlation between morning urine PCR, random urine PCR, and 24hUTP in different subgroups of patients, the results showed that morning urine PCR, random urine PCR, and 24hUTP in different subgroups were positively correlated, with correlation coefficients ranging from 0.50 to 0.99 (*P* < 0.05), and the correlation between random urine PCR and 24hUTP was higher than that of morning urine PCR in all subgroups. The correlation between morning urine PCR and random urine PCR and 24hUTP was found to be independent of eGFR in patients in different eGFR groups, which is consistent with previous reports [5], i.e., morning urine PCR or random urine PCR could be used to assess 24hUTP in patients with different stages of glomerulonephritis. The results of this trial were investigated, and the correlation between random urine PCR and 24hUTP was found to be higher than that of morning urine PCR. The reason for this may be the difference in urine concentration, osmolality, and urine creatinine content between morning urine and random urine. Even though the ratio form can correct for variations in urine concentration, there are individual differences, testing errors, and sampling errors, in addition to this part of the hydration, that make the test results between morning and random urine different [21]. The results of [7] showed that Alb levels had a little effect on the correlation between random urine PCR and 24 h urine protein, but the results of this study showed that the correlation between both morning urine PCR and random urine PCR and 24hUTP was lower when serum Alb was <30 g/L than when serum Alb was ≥30 g/L. In the present study, we analyzed different total cholesterol groups and showed that the correlation between morning urine and random urine PCR and 24hUTP was lower when total cholesterol was ≥6.0 mmol/L than when total cholesterol was <6.0 mmol/L. This is consistent with the study of [8], which may be due to the fact that most patients with total cholesterol ≥6.0 mmol/L had nephrotic syndrome as their primary disease. In the progression of nephrotic syndrome, patients develop hyperlipidaemia, profuse proteinuria, hypoproteinaemia, and oedema, especially when 24hUTP is ≥3.5 g, and the correlation between PCR and 24hUTP is significantly reduced, as confirmed by studies of glomerulonephritis.

In summary, this study demonstrates that morning urine PCR, random urine PCR, and 24hUTP all have good correlation, and the correlation between random urine PCR and 24hUTP is higher than that of morning urine PCR and establishes the prediction equation of morning urine PCR and random urine PCR on 24hUTP; this equation is more meaningful for assessing the condition as well as judging the prognosis of patients, because random urine PCR prediction equation. The random urine PCR prediction equation has a higher coefficient of determination than the morning urine PCR equation, so it is recommended that the random urine PCR prediction equation be used as an alternative to the 24hUTP test. However, this study also has shortcomings; as only some cases from a single centre were selected, the sample size was small and the subgroups were small, only one eGFR was considered in the renal function subgroup, and only one Alb was considered in the liver function subgroup [22, 23].

## 7. Conclusions

The use of monoclonal antibodies in the clinical treatment of FSGS has been gaining momentum in recent years as the research and application of this technology continue to advance. Currently, ofatumumab is one of the most promising monoclonal antibodies other than RTX for renal applications. As a humanised monoclonal antibody targeting CD20, ofatumumab does not recognise the same epitopes as RTX. In case reports, ofatumumab appears to be superior to RTX due to its lower adverse effects at higher doses. Therefore, its therapeutic efficacy and mechanism of action need to be further investigated. In addition, other monoclonal antibodies such as adalimumab, fresolimumab, and bleselumab are being explored for the treatment of FSGS.

## Figures and Tables

**Figure 1:** Correlation analysis of morning urine PCR with 24hUTP.

**Figure 2:** Correlation analysis of random urine PCR with 24hUTP.

**Figure 3:** ROC curves of morning urine PCR and random urine PCR predicting 24hUTP ≥ 0.5 g.

**Figure 4:** ROC curves of morning urine PCR and random urine PCR for predicting 24hUTP ≥ 1.0 g.

**Figure 5:** ROC curves of morning urine PCR and random urine PCR for predicting 24hUTP ≥ 3.5 g.

**Table 1:** General information about the study population.

Project	Numerical value

Age (years)	57.6±17.3
Male (cases (%))	107 (50.7)
Primary (cases (%))	176 (83.4)
24 hUTP (g)	1.9±1.6
24 h urine volume (ml)	1480±546
Morning urine PCR (g/g)	2.0±1.7
A1b (g/L)	33.7±8.4
eGFR [mL min^−1^(1.73 m^2^)^−1^]	54±43.3
Total cholesterol (mmol/L)	4.9±2.0
Glomerulonephritis 1	65 (30.81)
Glomerulonephritis 2	24 (11.37)
Glomerulonephritis 3	26 (12.32)
Glomerulonephritis 4	27 (12.8)
Glomerulonephritis 5	69 (32.7)

**Table 2:** Correlation between morning urine PCR, random urine PCR, and 24hUTP for different subgroups.

Group		Number of cases	Morning urine PCR (g/g)	Random urine PCR (g/g)	24hUTP (g)	*r*_1_	*r*_2_

Gender	Male	107	2.0±1.7	1.8±1.5	1.8±1.5	0.92	0.97
	Female	104	2.1±1.6	2.2±1.6	2.1±1.7	0.89	0.93
Age (years)	<45	43	1.4±1.2	1.5±1.3	1.5±1.2	0.91	±0.96
	45–60	81	1.8±1.5	2.0±1.6	1.9±.7	0.86	0.92
	>60	87	2.5±19	2.3±1.6	2.2±1.6	0.91	0.97
24 h urine volume (ml)	≤2000	174	2.2±1.7	2.1±1.6	2.0±1.6	0.91	0.95
	>2000	37	2.3±1.0	1.4±1.1	1.4±1.2	0.83	0.89
Pathogeny	Primary renal damage	176	1.5±1.7	1.8±2.0	1.2±1.6	0.71	0.82
	Secondary renal damage	35	1.7±2.2	1.5±2.3	1.7±2.5	0.96	0.99
eGFR [mL min^−1^(1.73 m^2^)^−1^]	≥90	65	0.4±0.3	0.5±0.4	0.4±0.4	0.68	0.71
	60–89	24	1.5±0.8	1.8±0.8	1.9±1.4	0.5	0.68
	30–59	26	2.6±2.0	2.6±2.0	2.4±2.0	0.95	0.99
	15–29	27	2.8±1.3	2.9±1.4	2.8±1.5	0.87	0.96
A1b (g/L)	<15	69	3.2±1.2	3.0±1.2	2.8±1.2	0.87	0.93
	<30	60	3.6±1.2	3.5±1.2	3.6±1.2	0.68	0.87
	≥30	151	1.4±1.4	1.4±1.3	1.3±1.2	0.91	0.95
Total cholesterol (mmol/L)	<6.0	148	1.4±1.4	1.5±1.3	1.3±1.3	0.92	0.95
	≥6.0	63	3.4±1.4	3.3±1.4	3.3±1.41	0.75	0.89

**Table 3:** Multiple linear regression analysis of morning urine PCR, random urine PCR, and 24hUTP.

Equation number	Independent variable	B	*P*	Coefficient of determination *R*^2^

Fang Cheng (1)	Morning urine PCR	0.793	<0.001	0.87
	Total cholesterol	0.124	<0.001	
	A1b	−0.177	<0.001	
	Constant	1.13	0.008	

Fang Cheng (2)	Morning urine PCR	0.856	<0.001	0.92
	Total cholesterol	0.132	<0.001	
	A1b	−0.092	0.001	
	Constant	0.369	0.265	

## Data Availability

The datasets used to support the findings of this paper are available from the corresponding author upon request.

## References

[1] Gunnarsson I., Sundelin B., Jónsdóttir T., Jacobson S. H., Henriksson E. W., van Vollenhoven R. F. (2007). Histopathologic and clinical outcome of rituximab treatment in patients with cyclophosphamide-resistant proliferative lupus nephritis. *Arthritis & Rheumatism*.

[2] Trachana M., Koutsonikoli A., Farmaki E., Printza N., Tzimouli V., Papachristou F. (2013). Safety and efficacy of rituximab in refractory pediatric systemic lupus erythematosus nephritis: A single-center experience of Northern Greece. *Rheumatology International*.

[3] Guiard E., Karras A., Plaisier E. (2011). Patterns of noncryoglobulinemic glomerulonephritis with monoclonal Ig deposits: Correlation with IgG subclass and response to rituximab. *Clinical Journal of the American Society of Nephrology*.

[4] Sfikakis P. P., Boletis J. N., Lionaki S. (2005). Remission of proliferative lupus nephritis following B cell depletion therapy is preceded by down-regulation of the T cell costimulatory molecule CD40 ligand: An open-label trial. *Arthritis & Rheumatism*.

[5] Hu X., Zhang J., Zhao Z., Wang S. (2015). Effect of rituximab on serum levels of anti-C1q antibodies and antineutrophil cytoplasmic autoantibodies in refractory severe lupus nephritis. *Hong Kong Journal of Nephrology*.

[6] Lindholm C., Börjesson-Asp K., Zendjanchi K., Sundqvist A. C., Tarkowski A., Bokarewa M. (2008). Longterm clinical and immunological effects of anti-CD20 treatment in patients with refractory systemic lupus erythematosus. *Journal of Rheumatology*.

[7] Atisha‐Fregoso Y., Malkiel S., Harris K. M. (2021). Phase II randomized trial of rituximab plus cyclophosphamide followed by belimumab for the treatment of lupus nephritis. *Arthritis & Rheumatology*.

[8] Fenoglio R., Sciascia S., Naretto C. (2020). Rituximab in severe immunoglobulin-A vasculitis (Henoch-Schonlein) with aggressive nephritis. *Clinical & Experimental Rheumatology*.

[9] Mendez L. M. G., Cascino M. D., Garg J. (2018). Peripheral blood B cell depletion after rituximab and complete response in lupus nephritis. *Clinical Journal of the American Society of Nephrology*.

[10] Ruggenenti P., Cravedi P., Chianca A. (2012). Rituximab in idiopathic membranous nephropathy. *Journal of the American Society of Nephrology*.

[11] Waldman M., Beck L. H., Braun M., Wilkins K., Balow J. E., Austin H. A. (2016). Membranous nephropathy: Pilot study of a novel regimen combining cyclosporine and rituximab. *Kidney international reports*.

[12] Nasr S. H., Sethi S., Cornell L. D. (2011). Proliferative glomerulonephritis with monoclonal IgG deposits recurs in the allograft. *Clinical Journal of the American Society of Nephrology*.

[13] Kodner C. (2016). Diagnosis and management of nephrotic syndrome in adults. *American Family Physician*.

[14] Barsolou J., John R., Bargman J. M. (2013). If it’s not one thing it’s another: Transformation of lupus nephritis. *CRAJ*.

[15] Leung A. K., Wong A. H., Barg S. S. (2017). Proteinuria in children: Evaluation and differential diagnosis. *American Family Physician*.

[16] Ravani P., Rossi R., Bonanni A. (2015). Rituximab in children with steroid-dependent nephrotic syndrome: A multicenter, open-label, noninferiority, randomized controlled trial. *Journal of the American Society of Nephrology*.

[17] Korte M. R., van Heerde M. J., de Man R. A., Betjes M. H. (2008). Rituximab for the treatment of glomerulonephritis in hepatitis C associated cryoglobulinaemia. *The Netherlands Journal of Medicine*.

[18] Hui D., Hladunewich M. A. (2019). Chronic kidney disease and pregnancy. *Obstetrics & Gynecology*.

[19] Zhengwan Z., Chunjiong Z., Hongbing L., Tao X. (2020). Multipath transmission selection algorithm based on immune connectivity model. *Journal of Computer Applications*.

[20] Bertsias G. K., Tektonidou M., Amoura Z. (2012). Joint European lagainst rheumatism and European renal association-European dialysis and transplant association (EULAR/ERA-EDTA) recommendations for the management of adult and paediatric lupus nephritis. *Annals of the Rheumatic Diseases*.

[21] Rosenstock J. L., Markowitz G. S. (2019). Fibrillary glomerulonephritis: An update. *Kidney international reports*.

[22] Yang Y., Yang L., Chen H., Yang J., Fan C. (2020). Risk factors of consumer switching behaviour for cross-border e-commerce mobile platform. *International Journal of Mobile Communications*.

[23] Luo Y., Ma J., Li C. (2020). Entity name recognition of cross-border e-commerce commodity titles based on TWs-LSTM. *Electronic Commerce Research*.

